The article "Affecting factors and seasonal effects on the continuous positive airway pressure adherence of patients with obstructive sleep apnea" was published in 2024. Journal: Heliyon.

# Affecting factors and seasonal effects on the continuous positive airway pressure adherence of patients with obstructive sleep apnea

**DOI:** 10.1016/j.heliyon.2024.e39840

**Published:** 2024-10-26

**Authors:** Jung Ju Lee, Bong Jin Jang, Daeho Kwon, Hyeyun Kim

**Affiliations:** a Sleep Medicine Research Center, Department of Neurology, College of Medicine, Catholic Kwandong University International St. Mary's Hospital, Incheon 22711, Republic of Korea; b Department of Medical Business Administration, Daegu Haany University, 201, Daegudae-ro, Gyeongsan-si 38610, Republic of Korea; c Department of Microbiology, College of Medicine, Catholic Kwandong University, Gangneung 25601, Republic of Korea

**Keywords:** Continuous positive airway pressure, Obstructive sleep apnea, Seasonal change, Apnea hypopnea index, Excessive daytime sleepiness, Insomnia

## Abstract

Continuous positive airway pressure (CPAP) is the preferred treatment for obstructive sleep apnea (OSA), but adherence remains challenging. This study identifies factors influencing CPAP adherence, including the impact of Korea's four distinct seasons. A retrospective study of 650 patients with OSA and prescribed with CPAP was conducted at a single institution from January 2018 to December 2020, and the patients' answers on various sleep questionnaires, demographic and polysomnographic data, and when and whether they returned the CPAP devices were collected and analyzed. The sample population was divided into when and whether the CPAP device was returned to the institution and the average daily use of the CPAP device. Results show that treatment failure is high in the first 12 weeks. Moreover, patients with more severe sleep apnea tended to have severe OSA-related clinical symptoms and are more likely to adhere to the treatment. In this study show that the seasons did not affect CPAP adherence because of indoor environmental factors. However, results show that other patient factors, such as BMI, AHI, RDI, daytime drowsiness, mood changes, and other OSA-related symptoms, have greater effects on CPAP adherence than seasonal change. Initial positive experience is important to adapt to the CPAP, and for this reason, more active intervention by sleep physicians during the initial CPAP adaptation is necessary.

## 1 Introduction

Obstructive sleep apnea (OSA) is a common sleep disorder characterized by abnormal and repetitive upper airway obstruction during sleep [1]. Recent global estimates suggest that nearly 1 billion adults worldwide suffer from OSA, representing approximately 36 % of the population aged 30–69 years [2]. In Korea, OSA prevalence was reported in 4.5 % of men and 3.2 % of women [3]. This sleep disorder worsens the quality of sleep and increases the risk of daytime sleepiness, reduced work performance, cognitive dysfunction, and cardiovascular disease [4]. Moreover, it is associated with cardiovascular diseases such as hypertension and myocardial infarction and increases the risk of diabetes, depressive disorder, glaucoma, Parkinson's disease, and infertility [[5], [6], [7], [8]]. Continuous positive airway pressure (CPAP) is the recommended treatment choice for OSA [9,10]. Because the effectiveness of treatment effect is determined by a patient's adherence to the treatment, one of the clinician's main roles here is to improve CPAP adherence. The adherence rate to CPAP treatment ranges from 28 % to 83 %, and similar results in Korea are reported with an adherence rate of around 40 % [11].

Given the significant health risks associated with untreated OSA, including increased cardiovascular and metabolic complications, improving CPAP adherence remains a crucial public health challenge [12]. Various factors may affect adherence to CPAP, including the severity of sleep apnea, patient characteristics and comorbidities, CPAP equipment, side effects of treatment, psychological factors, and socioeconomic considerations [13].

While these factors have been extensively studied, the potential influence of seasonal variation on CPAP adherence, particularly in countries with distinct seasons like Korea, remains largely unexplored. Understanding the impact of seasonal changes on CPAP use could provide valuable insights for optimizing treatment strategies and improving year-round adherence to CPAP therapy.

This study aimed to identify the factors, including seasonal variation, affecting the adherence to CPAP in a Korean population. By examining these influences, we hope to contribute to the development of more effective, personalized approaches to OSA management, ultimately improving patient outcomes and quality of life.

## 2 Materials and methods

### 2.1 Study design and participants

This retrospective study was conducted at a single institution from January 2018 to December 2020. The study population consisted of adults aged 20 years or older who were diagnosed with obstructive sleep apnea (OSA) through polysomnography (PSG), with an apnea-hypopnea index (AHI) of 5 or more events per hour. Only patients who were prescribed continuous positive airway pressure (CPAP) therapy and used it for at least two weeks were included in the study.

We excluded patients with central sleep apnea, those with incomplete medical records or CPAP usage data, and individuals unable to use CPAP due to medical conditions unrelated to OSA.

A total of 650 patients meeting these criteria were included in the study. As this was a retrospective analysis of all eligible patients over a three-year period, we did not perform a formal sample size calculation prior to data collection. However, a post-hoc power analysis revealed that this sample size was sufficient to detect a medium effect size (Cohen's d = .5) with 80 % power at a significance level of .05 for the main comparisons between groups.

This approach allowed us to clearly define the inclusion and exclusion criteria for our study population, while also addressing the issue of sample size and statistical power. By including all eligible patients over the specified time period, we aimed to maximize the representativeness of our sample within the constraints of a single-institution retrospective study.

Patient demographics were collected and analyzed, such as age, gender, body mass index (BMI), PSG data, and their answered sleep questionnaires for sleep and emotional statuses. The questionnaires included a daytime sleepiness evaluation using the Epworth Sleepiness Scale (ESS) [14], Stanford Sleepiness Scale [15], and STOP-Bang [16] to evaluate sleep apnea and the Hospital Anxiety and Depression Scale (HADS) [17].

For scoring obstructive sleep apnea (OSA), we adhered to the American Academy of Sleep Medicine (AASM) 2012 scoring manual for sleep and associated events. In our study, apneas were identified as a 90 % or greater decrease in airflow lasting at least 10 s. Hypopneas were scored using the recommended AASM definition, which is a 30 % or greater decrease in airflow for at least 10 s, associated with either a 3 % or greater oxygen desaturation or an arousal.

Our polysomnography (PSG) data acquisition and analysis were conducted using the NOX A1 PSG system (Nox Medical, Reykjavik, Iceland). This comprehensive sleep diagnostic system allowed us to record a wide range of physiological parameters. We utilized the Noxturnal software, which is specifically designed for use with the NOX A1 system, for data analysis and interpretation.

The NOX A1 system enabled us to record electroencephalogram (EEG) with leads at F3-M2, F4-M1, C3-M2, C4-M1, O1-M2, O2-M1, electrooculogram (EOG), chin and bilateral anterior tibialis electromyogram (EMG), and electrocardiogram (ECG). We also monitored airflow using both a nasal pressure transducer and an oronasal thermistor, respiratory effort via RIP (Respiratory Inductance Plethysmography) belts for thorax and abdomen, oxygen saturation using pulse oximetry, body position, and snoring sounds.

Patients in our study were prescribed one of three CPAP devices: the ResMed AirSense 10 AutoSet, the Philips Respironics DreamStation Auto, or the Fisher & Paykel SleepStyle Auto. All of these devices were configured to operate in auto-titrating mode, with a pressure range set between 4 and 20 cmH2O. All CPAP devices were equipped with integrated humidifiers. The humidification settings were adjustable and patients were instructed on how to modify these settings for optimal comfort.

In addition, the seasons were divided into spring (March to May), summer (June to August), autumn (September to November), and winter (December to February). The seasonal factor was based on when the CPAP device was returned to the institution, while the treatment failure rate was based on whether the CPAP device was returned at all. Good and poor treatment adherence was measured according to the average daily use of the CPAP device, wherein poor adherence denoted <4 h of use per day and good adherence denoted >4 h of use per day.

This study was conducted after review and approval by the Institutional Review Board (IRB No. IS20OISE0059, 2020/9/14) of International St. Mary's Hospital, Catholic Kwandong University.

### 2.2 Statistical analyses

Factors influencing CPAP failure were analyzed by dividing them into two groups: those that continued treatment (CPAP Keep) and those who failed to adhere to the CPAP treatment (CPAP Fail). The classification standard was based on the patient's use of the CPAP device in hours per day, where the cut-off point was an average of 4 h per day of use. The participants were further divided into “Good Adherence” and “Poor Adherence” groups based on the cut-off point. SPSS 21.0 (SPSS for Windows, SPSS Inc, USA) was used for data analysis. Specifically, the comparison between the two groups was analyzed using the paired *t*-test. Binary logistic regression was used to analyze the influencing factors to CPAP because the dependent variable (CPAP) is a nominal scale. Descriptive information was presented as a percentage or as mean ± standard deviation. All *p*-values <.05 were considered statistically significant.

## 3 Results

### 3.1 Descriptive demographics

A total of 650 patients were diagnosed with OSA and prescribed CPAP for 3 years, from January 1, 2018, to December 31, 2020. In particular, there were 149 patients (22.9 %) in the spring, 191 patients (29.4 %) in the summer, 154 patients (23.7 %) in the fall, and 156 patients (24 %) in the winter. The frequency of CPAP prescriptions did not differ by season. Of the 650 enrolled patients diagnosed with OSA, 278 patients (42.7 %) failed the CPAP therapy.

### 3.2 CPAP treatment failure according to CPAP use

CPAP failure was analyzed in 4-week intervals, resulting in a high return rate within the first 12 weeks of treatment and a decrease after week 13 (Table 1 and Fig. 1).

**Table 1:** CPAP treatment failure rate according to the period of use (weekly).

Period of Use (weeks)	Number of Returns	Period of Use (weeks)	Number of Returns	Period of Use (weeks)	Number of Returns
1–4	30	37–40	21	73–76	18
5–8	68	41–44	22	77–80	16
9–12	63	45–48	25	81–84	25
13–16	53	49–52	15	85–88	16
17–20	19	53–56	23	89–92	15
21–24	22	57–60	25	93–96	19
25–28	24	61–64	21	97–100	15
29–32	21	65–68	21	101–104	17
33–36	20	69–72	22	Total	275

**Fig. 1:** CPAP treatment failure rate according to the period of use (weekly).

### 3.3 The differences between CPAP fail and CPAP keep groups

In the group CPAP Keep group, BMI was higher (p = 0.009) than in the group that returned the CPAP Fail group. In addition, the CPAP Keep group's AHI (47.33/h) and respiratory disturbance index (RDI) (47.88/h) were significantly more severe than the CPAP Fail group's AHI of 41.17/h and RDI of 47.88/h (p < 0.001). Table 2 presents the differences in characteristics between the CPAP Fail and Keep groups according to demographic data and polysomnographic findings.

**Table 2:** The differences between CPAP return and keep groups according to demographic data and the results from polysomnographic findings.

Characteristic	CPAP Fail (n = 278)	CPAP Keep (n = 372)	*p*
Female (n,%)	66,48.5 %	70,51.5 %	
Male (n,%)	212,41.2 %	302, 58.8 %	
Age (yrs)	52.02 (_±_13.72)	49.15 (_±_12.88)	
BMI (kg/m^2^)	26.76 (_±_4.83)	27.79 (_±_5.17)	.009∗
TST (minutes)	375.83 (_±_57.02)	371.97 (_±_52.15)	.376
N1 (%)	32.32 (_±_22.49)	32.74 (_±_16.47)	.791
N2 (%)	42.99 (_±_18.12)	39.93 (_±_10.71)	.012
N3 (%)	9.80 (_±_7.08)	10.05 (_±_7.27)	.654
REM (%)	18.34 (_±_8.14)	17.27 (_±_6.38)	.072
Total wake time (minutes)	14.08 (_±_22.66)	11.71 (_±_9.72)	.103
WASO (minutes)	59.00 (_±_55.51)	51.73 (_±_43.15)	.071
Latency to sleep (minutes)	10.95 (_±_17.41)	9.52 (_±_10.26)	.222
Latency to REM onset (minutes)	116.51 (_±_78.03)	114.62 (_±_74.18)	.756
Sleep efficiency (%)	84.59 (_±_11.92)	85.85 (_±_10.17)	.156
AHI (per hour)	41.17 (_±_21.04)	47.33 (_±_23.02)	<.001∗
RDI (per hour)	41.93 (_±_20.70)	47.88 (_±_22.78)	<.001∗
PLMS (per hour)	5.75 (_±_16.02)	4.60 (_±_14.28)	.344

BMI, Body mass index; TST,Total Sleep Time; N, Non-REM stage; REM, Rapid eye movement; WASO, wakefulness after sleep onset; AHI, Apnea hypopnea index; RDI, respiratory disturbance index; PLMS, Periodic limbs movement during sleep.

The daytime sleepiness based on the ESS and anxiety score according to the HADS were higher in the CPAP Keep group. The STOP-Bang score, a screening tool for snoring and sleep apnea, was higher in the CPAP Keep group. The characteristics of the CPAP Fail and Keep groups according to sleep questionnaires are shown in Table 3.

**Table 3:** The differences between CPAP return and keep groups according the results from questionnaires.

Questionnaire	CPAP Fail (n = 278)	CPAP Keep (n = 372)	*p*
Epworth Sleepiness Scale	8.87 (±4.71)	10.57 (±5.07)	.000∗
Stanford Sleepiness Scale	3.13 (±1.49)	2.97 (±1.43)	.174
HAD_Anxiety	8.34 (±4.37)	7.55 (±4.10)	.020∗
HAD_Depression	6.50 (±4.04)	5.96 (±3.72)	.083
ISI	12.37 (±6.32)	12.80 (±6.09)	.383
STOP-BANG	4.20 (±1.34)	4.48 (±1.30)	.009∗

HAD, Hospital Anxiety Depression; ISI, Insomnia severity index.

### 3.4 The differences between good adherence and poor adherence of CPAP

The CPAP usage time was calculated as the average daily time, where the Good Adherence group followed through with the CPAP for >4 h per day and the Poor Adherence group complied with the treatment for <4 h per day. The affecting factors in both groups are shown in Table 4. The proportion of non-rapid eye movement (non-REM) sleep stage 3 (N3) was lower in the Good Adherence group than the Poor Adherence group. However, the AHI and RDI, indicators of sleep apnea severity, were significantly higher in the Good Adherence group than the Poor Adherence group (*p* = 0.008). Moreover, in Table 5, the STOP-Bang score, a screening tool for snoring and sleep apnea, was higher in the Good Adherence group (*p* = 0.045). The severity of anxiety/depression, according to the HADS, was more severe in the Poor Adherence group than the Good Adherence group (*p* < 0.001).

**Table 4:** The affecting factors attributing to adherence of CPAP.

Characteristic	Poor adherence (n = 388)	Good adherence (n = 262)	*p*
Female (n,%)	81 (59.6 %)	55 (40.4 %)	
Male (n,%)	307 (59.7 %)	207 (40.3 %)	
Age (years)	49.37 (_±_13.36)	51.88 (_±_13.12)	
BMI (kg/m^2^)	27.30 (_±_5.52)	27.43 (_±_4.28)	.754
TST (minutes)	437.94 (_±_36.53)	435.75 (_±_27.39)	.411
N1 (%)	37.44 (_±_17.94)	37.25 (_±_15.61)	.668
N2 (%)	31.99 (_±_20.66)	33.40 (_±_16.99)	.361
N3 (%)	42.28 (_±_16.34)	39.69 (_±_10.85)	.025∗
REM (%)	10.24 (_±_7.08)	9.49 (_±_7.32)	.192
Total wake time (minutes)	17.94 (_±_7.49)	17.41 (_±_6.74)	.356
WASO (minutes)	13.05 (_±_19.63)	12.24 (_±_10.52)	.543
Latency to sleep (minutes)	54.86 (_±_49.83)	54.81 (_±_47.61)	.989
Latency to REM onset (minutes)	117.38 (_±_77.94)	112.53 (_±_72.53)	.426
Sleep efficiency (%)	85.27 (_±_11.06)	85.37 (_±_10.83)	.909
AHI (per hour)	42.78 (_±_22.03)	47.53 (_±_22.66)	.008∗
RDI (per hour)	43.44 (_±_21.73)	48.14 (_±_22.38)	.008∗
PLMS (per hour)	5.93 (_±_17.27)	3.84 (_±_10.87)	.081

BMI, Body mass index; TST, Total Sleep Time; N, Non-REM stage; REM, Rapid eye movement; WASO, wakefulness after sleep onset; AHI, Apnea hypopnea index; RDI, respiratory disturbance index; PLMS, Periodic limbs movement during sleep.

**Table 5:** Differences between poor and good adherence to CPAP treatment according to questionnaire answers.

Questionnaire	Poor adherence (n = 388)	Good adherence (n = 262)	*p*
Epworth Sleepiness Scale	9.62 (±5.09)	10.18 (±4.82)	.166
Stanford Sleepiness Scale	3.12 (±1.41)	2.92 (±1.52)	.082
HAD_Anxiety	8.45 (±4.29)	7.05 (±4.00)	<.001∗
HAD_Depression	6.61 (±3.93)	5.56 (±3.70)	<.001∗
ISI	12.92 (±6.13)	12.18 (±6.25)	.135
STOP-BANG	4.28 (±1.36)	4.49 (±1.25)	.045

HAD, Hospital Anxiety Depression; ISI, Insomnia severity index.

## 4 Discussion

As factors that may affect adherence to CPAP, the severity of sleep apnea, the patient's characteristics and comorbidities, CPAP equipment, side effects of CPAP treatment, psychological underlying, and socioeconomic factors of the patients were considered [18]. Among the factors, it was expected that there would be seasonal influences based on the four distinct seasons as in Korea, but no research has been done on this to date. A similar study in Japan [19] found longer sleeping times in winter, resulting in higher treatment compliance and lower compliance in the spring when allergic rhinitis worsens. However, it was found that seasonal factors did not affect CPAP adherence. Notably, countries with shared health insurance contracts felt higher out-of-pocket costs at the beginning of the year and lowered compliance. Moreover, it noted that only a few reports of small groups in domestic and overseas studies on seasonal factors had been published.

A German study proposed no difference in temperature and humidity of the use environment depending on the season because air-conditioning control is possible in the environment of users’ homes where the CPAP device is used [20]. In addition, seasonal allergic rhinitis could be a negative factor for CPAP adherence. However, humidification could be adjusted in newer CPAP devices. Increasing the level of humidification in CPAP devices may resolve the uncomfortable dryness due to seasonal allergic rhinitis [20]. In contrast, another study found that allergic rhinitis did not increase the risk of sleep apnea [21]. Therefore, the results of previous studies suggesting that exacerbation of spring allergic rhinitis may have affected CPAP adherence are controversial.

Studies on seasonal changes in CPAP use are scarce, and more research is needed to reach a clear conclusion. Because Korea's environment is characterized by distinctive changeable seasons, especially with severe pollen issues in the spring and the hot and humid summers, the results of this study should be treated in earnest. Many patients struggled to use a CPAP mask in the summer and complained about its difficulty due to sweating. However, as shown in the results of this study, the summer months showed no negative effect on adherence to CPAP treatment. A patient's complaints about the difficulty of using a CPAP device according to seasonal changes are frequently encountered in the clinical field, so the complaints about seasonal effects should not be ignored. However, it should be recognized that other patient factors, such as BMI, AHI, RDI, daytime drowsiness, mood changes, and other OSA-related symptoms, have greater effects on CPAP adherence than seasonal change.

Obesity and OSA are interrelated as obesity is a known risk factor for OSA [22]. Proper therapy for OSA is a recommended treatment strategy in the treatment of obesity. However, a study showed that CPAP use for OSA treatment does not control obesity [23]. Although many studies on the causal relations and treatment mechanism of obesity and OSA, it is difficult to simplify their relationship and treatment effects. In the current study, a high BMI was a positive factor in CPAP adherence. Because a patient's voluntary and active behavioral attitude is necessary, this result could be interpreted as being more active in CPAP treatment in patients with obesity. However, further studies between obesity and CPAP adherence are required to clarify this relationship.

In this study, CPAP adherence was closely related to the severity of sleep apnea with increased AHI/RDI. Those with severe sleep apnea are more active in CPAP treatment and adapt well to the results of previous studies [18,24,25]. The more severe the OSA, the higher the number of comorbidities, and the higher the frequency of clinical symptoms such as daytime sleepiness [[26], [27], [28]]. The OSA comorbidity was not included in this study's analysis. However, upon reviewing previous studies and based on this study's high levels of ESS and anxiety levels, it is considered that active behavior on CPAP treatment in patients with more frequent comorbidities could be addressed in future studies.

A lower proportion of N3 stage sleep indicates more severe sleep apnea, which was found in the Good Adherence group of this study. Therefore, the low proportion of N3 stage sleep was related to the severity of OSA, which the high adherence to CPAP treatment could explain. Although not analyzed in this study, it has been reported that the proportion of N3 stage, slow-wave sleep also showed rebound increase when the OSA is successfully treated with good adherence to CPAP therapy [29].

In Korea, CPAP therapy is covered by national health insurance after successful initial adherence to the treatment for three months. For this reason, it appears that the exact point of initial adherence in this study was different based on the 12 weeks. Moreover, it was difficult to ascertain pure initial adherence regardless of health insurance issues. Although it is not related to the national health insurance system, several studies already reported that early compliance is important [30,31], and this study also provides similar results. Thus, initial positive experience is important to adapt to the CPAP, and for this reason, more active intervention by sleep physicians during the initial CPAP adaptation is necessary.

This study has several limitations that should be considered when interpreting the results. Firstly, as a single-center, retrospective study, our findings may not be fully generalizable to other populations or healthcare settings. The retrospective nature of the study also limits our ability to control for all potential confounding factors that might influence CPAP adherence.

Secondly, while we examined seasonal effects, we did not have detailed information on indoor environmental factors such as bedroom temperature and humidity, which could potentially impact CPAP use. Future prospective studies incorporating these factors could provide more comprehensive insights into environmental influences on CPAP adherence.

Thirdly, our study relied on self-reported questionnaire data for assessing symptoms and quality of life measures. These subjective measures may be influenced by recall bias or other factors that could affect their accuracy. Fourthly, while we had data on CPAP usage, we did not have detailed information on mask type or humidification settings, which could also influence adherence. Including these factors in future studies could provide a more nuanced understanding of CPAP adherence determinants. Lastly, our follow-up period was limited to the duration of the study. Longer-term follow-up studies could provide valuable information on sustained CPAP adherence patterns and their relationship to seasonal variations over extended periods. While we collected data on comorbidities and medications, we did not have detailed information on the severity or duration of these conditions, or on medication dosages and adherence. Future studies could benefit from a more comprehensive assessment of these factors and their potential impact on CPAP adherence.

Despite these limitations, our study provides important insights into the factors influencing CPAP adherence in a Korean population, including the potential role of seasonal variations. These findings can inform future research directions and clinical strategies for improving CPAP adherence.

## 5 Conclusion

Seasonal variation did not affect CPAP adherence. The severity of OSA, the frequency of OSA-related clinical symptoms, and high BMI are positive factors for good adherence to CPAP treatment.

## CRediT authorship contribution statement

**Jung Ju Lee:** Writing – original draft, Visualization, Validation, Software, Project administration, Methodology, Funding acquisition, Formal analysis, Data curation, Conceptualization. **Bong Jin Jang:** Writing – original draft, Visualization, Validation, Software, Project administration, Methodology, Funding acquisition, Formal analysis, Data curation, Conceptualization. **Daeho Kwon:** Writing – review & editing, Writing – original draft, Validation, Project administration, Methodology, Formal analysis, Data curation, Conceptualization. **Hyeyun Kim:** Writing – review & editing, Writing – original draft, Validation, Supervision, Software, Resources, Project administration, Methodology, Investigation, Funding acquisition, Formal analysis, Data curation, Conceptualization.

## Informed consent statement

Not applicable.

## Institutional Review Board statement

Not applicable.

## Funding

None.

## Declaration of competing interest

The authors declare that they have no known competing financial interests or personal relationships that could have appeared to influence the work reported in this paper.
